The article "Snapping Sternoclavicular Joint" was published in 2023. Journal: Cureus.

# Snapping Sternoclavicular Joint

**DOI:** 10.7759/cureus.38557

**Published:** 2023-05-04

**Authors:** Paul V Romeo, Aidan G Papalia, Neil Gambhir, Stuart T Styles, Mandeep S Virk

**Affiliations:** 1 Department of Orthopedic Surgery, New York University (NYU) Langone Orthopedic Hospital, New York, USA; 2 Department of Orthopedic Surgery, Somers Orthopedic Surgery and Sports Medicine Group, Carmel Hamlet, USA

**Keywords:** sternoclavicular, clavicular pathology, diarthrodial joint, snapping sternoclavicular joint, sternoclavicular joint

## Abstract

Snapping sternoclavicular joint (SCJ) is a rare presentation in the SCJ. We present a case report detailing the presentation and treatment of unilateral snapping SCJ in a 14-year-old male patient. Clinical findings included the subluxation of the medial end of the clavicle in the anterior-posterior direction following a specific maneuver by the patient that involved repetitive external rotation with the arm in horizontal abduction. Dynamic ultrasound demonstrated an asymmetric widening of the right sternoclavicular joint in the neutral position with a pronounced subluxation in provocative positioning. At 3.5-year follow-up, he continued to remain pain-free without static deformity of the SCJ. Snapping SCJ is a benign phenomenon that does not require any intervention and is not associated with ligament laxity.

## Introduction

The instability of the sternoclavicular joint (SCJ) is a rare presentation and most commonly seen as a consequence of trauma, although reports exist detailing this entity as a sequela of connective tissue disorders, congenital malformations, or arthritis of the SCJ [1-7]. Atraumatic spontaneous SCJ subluxation is often bilateral and more commonly reported in females and has an association with generalized ligamentous laxity [1-4,8,9]. Though generally painless and self-reducible, the uncomfortable sensation of subluxation and the associated deformity can cause a great level of concern for patients and the providers taking care of them [1]. Reports of surgical treatment have been described for atraumatic subluxations with mixed results [4,8].

Unilateral SCJ subluxation and reduction, i.e., snapping SCJ, without underlying ligament laxity and without traumatic cause are unreported. We present a case of a 14-year-old patient with no history of trauma or underlying ligamentous laxity, who was treated nonoperatively for snapping SCJ. Herein, we discuss the clinical findings, diagnostic considerations, nonoperative treatment, and outcomes at a 3.5-year follow-up.

## Case presentation

The index patient is a 14-year-old right-hand-dominant male who presented with several weeks of right medial clavicle prominence near the sternum that was first noticed while flat barbell bench pressing. A painless click or snap was felt at the right SCJ when the prominence would appear. He noted that the prominence would self-reduce when his right arm was adducted to his side. The patient denied any recent trauma and had a noncontributory surgical and medical history. The patient was prompted to see an orthopedic surgeon out of concern for complications that could arise given his participation in recreational contact sports (ice hockey).

The physical examination of the SCJ revealed no obvious static deformity or subluxation of the SCJ with the arm in a neutral position by his side. However, the patient was able to anteriorly subluxate and reduce the medial end of the clavicle during a repetitive external rotation maneuver with the arm in horizontal abduction (Figure 1).

**Figure 1:** Anteriorly Subluxed Right Sternoclavicular Joint A: subluxed right sternoclavicular joint

The patient had normal shoulder range of motion with no neurological deficits. The Beighton score was 0, indicative of no ligament laxity [10]. Anterior-posterior X-ray radiographs demonstrated no deformity or additional pathology. Dynamic ultrasound performed in the clinic demonstrated an asymmetric widening and a pronounced anterior subluxation of the SCJ with the arm abducted (Figure 2 and Figure 3).

**Figure 2:** X-Ray: Anterior-Posterior View Red circle: right sternoclavicular joint

**Figure 3:** X-Ray: Anterior-Posterior View, 40 Degrees Cephalad Red circle: right sternoclavicular joint

The contralateral SCJ was normal and did not have snapping. Given the atraumatic and painless nature of subluxation, the patient was educated about this being idiopathic snapping SCJ and prescribed physical therapy aimed at rotator cuff and scapular stabilizer muscle strengthening. He was allowed to return to contact sports and other sporting activities. At 3.5-year follow-up, the patient continues to have painless snapping of the SCJ and no static deformity while also participating in competitive baseball and ice hockey (Table 1).

**Table 1:** Patient-Reported Outcomes at 3.5-Year Follow-Up PROMIS:Patient-Reported Outcome Measurement Information System [11,12]

	3.5-Year Follow-Up
PROMIS Upper Extremity	61
PROMIS Pain Interference	38.7
PROMIS Pain Intensity	30.7
American Shoulder and Elbow Surgeons Score	100
Visual Analog Score Pain Scale	0

## Discussion

In this report, we describe the natural history of a rare presentation of snapping SCJ. At 3.5-year follow-up, the patient continued to participate in contact sports without pain or any static deformity.

Gleason described a case of bilateral, spontaneous, anterior dislocation of the SCJ that occurred to a 20-year-old combat soldier. The figure-of-eight brace was attempted but deemed unsuccessful and abandoned for more conservative therapy without immobilization. Additional physical examination findings revealed the hyperlaxity of the patient’s wrists, knees, and ankles [2]. Echlin and Michaelson described a case of a 14-year-old female swimmer who experienced recurrent bilateral SCJ subluxation during active and passive abduction with forward flexion [3]. She had underlying ligament hyperlaxity affecting multiple joints. The patient elected for nonoperative treatment with activity modification and had a good result [3]. Sadr and Swann described 22 patients, 20 of whom were female and the majority middle-aged, with spontaneous anterior subluxation of the medial end of the clavicle. All patients were treated with analgesia and reassurance, which returned favorable outcomes [1]. Similarly, Kiel et al. noted that the most common patients for atraumatic SCJ subluxation were females with ligamentous laxity and multidirectional instability [5]. In contrast to the aforementioned studies, our patient had atraumatic snapping SCJ (subluxation and spontaneous reduction) with no underlying ligamentous laxity. Furthermore, dynamic ultrasound demonstrated no underlying ligament tears, ruling out the remote history of missed trauma.

Snapping SCJ is a benign painless condition and does not require surgical treatment. Although operative treatment for symptomatic anterior SCJ subluxation has been reported, as demonstrated by Rockwood and Odor, surgery predisposes patients to an increased propensity for complications [8]. Of the 37 patients they investigated, eight underwent surgical procedures with three requiring additional clavicular resections, one of whom suffered from thoracic outlet syndrome necessitating complete clavicular excision [8]. Hirsiger et al. reported outcomes in four patients who underwent rotational corrective osteotomy of the medial clavicle for chronic, symptomatic anterior subluxation of the SCJ [4]. However, there was a high incidence of complications including plate removal, plate failure, residual subjective or objective instability, and palpable crepitus, some of which required revision surgery [4]. Additional studies on the efficacy of operative measures for symptomatic SCJ instability and subluxation have found that surgery can provide pain relief but the results are unpredictable and associated with complications [4,9,13]. It is important to identify benign snapping SCJ and differentiate it from painful symptomatic SCJ instability (static subluxation or dislocation) because snapping SCJ does not require surgical treatment as shown in our case report.

Painless snapping has been described previously as a benign phenomenon in several synovial joints (the hip, scapula, knee, ankle, and elbow) and can have extraarticular or intraarticular etiology of the snapping sound. Painless snapping in the SCJ is an unusual phenomenon and is probably related to its unique anatomy. The SCJ is a diarthrodial joint with a range of motion limited to 35 degrees of anterior-posterior flexion and extension [3,5-7]. There are no tendons that cross the SCJ, and its primary stability is provided by the rigid posterior capsular ligaments [1,6]. Our patient denied any antecedent trauma, had no underlying generalized ligament laxity, and had a painless presentation of his symptoms, which required observation and education only and makes this case report unique in addition to reporting the rarity of this presentation in the SCJ.

## Conclusions

Sternoclavicular joint pathology has been detailed previously in patients with a predisposition, namely, females and those with ligamentous hyperlaxity and preceding trauma. However, as demonstrated with our patient here, snapping SCJ can present as a benign, rare presentation that may occur idiopathically with no preceding trauma or predisposition. For patients presenting with painless idiopathic cases, surgical intervention may not be warranted. Furthermore, it is important to note that this condition is not necessarily associated with generalized ligamentous laxity.

## References

[1] Sadr B, Swann M (1979). Spontaneous dislocation of the sterno-clavicular joint. Acta Orthop Scand.

[2] Gleason BA (2006). Bilateral, spontaneous, anterior subluxation of the sternoclavicular joint: a case report and literature review. Mil Med.

[3] Echlin PS, Michaelson JE (2006). Adolescent butterfly swimmer with bilateral subluxing sternoclavicular joints. Br J Sports Med.

[4] Hirsiger S, Hasler A, Fürnstahl P, Gerber C (2019). Chronic anterior sternoclavicular instability: technique and results of corrective clavicular osteotomy. J Shoulder Elbow Surg.

[5] Kiel J, Ponnarasu S, Kaiser K (2022). Sternoclavicular joint injury. StatPearls.

[6] Dhawan R, Singh RA, Tins B, Hay SM (2018). Sternoclavicular joint. Shoulder Elbow.

[7] Garcia JA, Arguello AM, Momaya AM, Ponce BA (2020). Sternoclavicular joint instability: symptoms, diagnosis and management. Orthop Res Rev.

[8] Rockwood CA Jr, Odor JM (1989). Spontaneous atraumatic anterior subluxation of the sternoclavicular joint. J Bone Joint Surg Am.

[9] Nettles JL, Linscheid RL (1968). Sternoclavicular dislocations. J Trauma.

[10] Malek S, Reinhold EJ, Pearce GS (2021). The Beighton score as a measure of generalised joint hypermobility. Rheumatol Int.

[11] Alben MG, Gordon D, Gambhir N (2023). Minimal clinically important difference (MCID) and substantial clinical benefit (SCB) of upper extremity PROMIS scores following arthroscopic rotator cuff repairs. Knee Surg Sports Traumatol Arthrosc.

[12] Romeo PV, Papalia AG, Alben MG (2023). Prognostic factors associated with improvements in patient-reported outcomes in idiopathic adhesive capsulitis. JSES Int.

[13] Guan JJ, Wolf BR (2013). Reconstruction for anterior sternoclavicular joint dislocation and instability. J Shoulder Elbow Surg.

